RETRACTED

# Art Painting Image Classification Based on Neural Network

**DOI:** 10.1155/2022/3119604

**Published:** 2022-07-04

**Authors:** Xiaodong Liu

**Affiliations:** Academy of Fine Arts, Linyi University, Linyi, Shandong 276000, China

## Abstract

Neural network (NN) is among the most important and vital form of artificial intelligence which are utilized for the classification of data, information, or images. Moreover, NN has been extensively utilized in various research domains throughout the world, and it is because of overwhelming properties. Painting is a form formed by China's long history and culture, and a large number of paintings reflect the living conditions of China in different periods, which is of great value to the development of China's culture. Image classification has become a key research content in the field of image in the stage of rapid development of information technology, and the content of art painting image classification has also developed rapidly. At present, most traditional image classification methods are formed on the basis of shallow structure learning algorithm, and there are many types of image features that can be extracted, but some features will be lost when extracting, and we need to master the basic painting knowledge. As a result, this extraction process is not general, which explains why traditional Chinese art picture classification is not ubiquitous. The fast development of big data technology and neural network algorithms in recent years has the potential to speed up the categorization of art painting images. As a result, this research investigates the use of neural networks to classify art painting images. The painting image classification method based on artistic style is used to determine the styles of distinct creative works, and the painting image classification algorithm based on saliency is then used to categorize the picture semantics. Finally, a dataset for testing the categorization impact of art painting pictures is developed. The results show that the neural network algorithm can significantly improve the classification effect of art painting images with higher accuracy.

## 1. Introduction

Artificial intelligence is the branch of computer science, which is focused how the electronics and machines are designed or modified such that these are capable to operate in a smart and intelligent way just like human beings do in the day-to-day activities. However, AI is further classified or divided into various branches such as neural network, deep learning, natural language process, and computer vision; among these, neural network is based on the idea of neurons which are basically the most vital factor of the human brain. Additionally, classification is utilized to effectively divide data values into the respective classes or groups which are based on certain threshold values and are based on the application parameter and problem domains. For example, classification of images could be based on high quality or medium or low-quality images. Additionally, it could be based on the size of the images as well such as small and large images, respectively. These classification models have applications or could be used in the different areas such as large dataset, classification of images. With the rapid development of digital images, more and more scholars began to study the field of image classification [1]. Art painting image classification is the main part of China's traditional culture. Through in-depth analysis, art painting image classification is conducive to the promotion of traditional culture, and the coverage is more abstract. Therefore, a large amount of professional knowledge should be used for feature extraction [2]. Because most of the traditional feature classification methods are completed on the basis of the shallow structure learning algorithm, only some image features can be extracted, which will also lead to the loss of some image features, resulting in many obstacles to the image classification of art painting in China [3].

RETRACTED

The most critical part of image classification is painting classification. This paper uses the neural network algorithm to train data by using multihidden layer network model, so as to more accurately express data features and improve the accuracy of classification results [4]. Therefore, it is feasible to use the neural network algorithm in the study of art painting image classification.

The main innovations in the research process of this paper are as follows: (1) this paper first describes in detail the concept of artificial neural network, the process of image classification calculation, and the process of convolution neural network image classification algorithm, which is taken as an important theoretical and algorithm basis for art painting image classification based on neural network. (2) Through the painting image classification algorithm based on art style to analyze and deal with the problem of painting image art style, calculate the similarity of each art painting image, then establish the painting image classification algorithm based on significance to calculate the image semantic classification, and complete the image classification analysis combined with the two algorithms.

The rest of the paper is arranged as given in the following paragraph.

Existing studies or work that is linked or related to the worked carried out in this paper is reported in Section 2. It is important to note that these schemes are presented along with their capacity in resolving an issue and what are the problems linked with it. NN-based classification of art painting images is presented in section three of the paper where we have started with brief introduction of the artificial intelligence and NN. Artistic painting image classification based on the neural network, which is the main contribution of this paper, is presented in section four of the paper. Results of the experimental setup is presented in Section 5 which is followed by the summarized form of the paper, i.e., conclusion.

RETRACTED

## 2. Related Work

With the continuous improvement of computer image processing technology, more and more people put forward higher demand for art works. Domestic and foreign experts have also deeply studied the field of image classification at home and abroad and achieved many remarkable results [5]. Hua et al. selected Dunhua murals and Oriental murals for research, analyzed the artistic style attributes of painting works, formulated the similarity rules of artistic style, and classified the artistic style of works by calculating the similarity coefficient between images [6]. Tesoro proposed an image semantic classification algorithm based on saliency, which uses the decomposition low rank matrix algorithm to reasonably divide the main areas of image semantics, effectively avoid the problem of painting semantics, and has become one of the commonly used methods in painting image semantic classification [7]. Hastings et al. proposed a way to evaluate the aesthetic visual quality and built a painting image visual quality model based on the designed local feature and global feature extraction method, so as to classify low vision and high visual quality paintings [8]. Knoos et al. deeply studied the traditional Chinese cultural painting images and formulated the classification method of Chinese painting images based on color features and texture features [9]. Alashari et al. proposed that for the extraction of texture features and color histogram on painting images, support vector machine (SVM) is selected as the classifier to accurately classify Chinese traditional painting images [10]. In the field of image classification and recognition, convolutional neural network has achieved remarkable results, but it is still in the early stage of research in painting image classification. Lu et al. used convolutional neural network to learn and recognize natural images that can improve the recognition effect of painting images [11]. Tian et al. proposed to automatically extract the stroke features of Chinese ink painting by using the convolution neural network based on mixed sparse. The classification effect obtained by classifying according to each author is ideal [12]. Xu and other experts proposed to use Sobel edge detection algorithm to locate the style features of ink painting and realize the automatic classification of various artist styles based on histogram features [13]. Weng et al. classified the painting style and painters based on the texture and color features of Chinese painting [14]. Meng et al. identified the authenticity of each author's painting image according to the stroke characteristics of each author's painting style by analyzing the characteristics of painting art style [15]. Liu et al. compared the sparse granularity and sparsity between freehand brushwork and fine brushwork, and classified the two types of paintings by edge size [16]. Xiao et al. analyzed the influence of convolution neural network structure width, convolution kernel size, and training sample number on classification results, optimized network structure and parameters, and formulated painting image classification algorithm based on convolution neural network [17].

RETRACTED

## 3. Image Classification Based on Neural Network

Classification is defined as the process of separating various objects in to the classes or groups where probability of similarity indexes between elements of a particular group is very high, i.e., it is high likely that elements or objects or data belong to a group which will be similar than other data values belonging to other groups or classes. ANN is a mechanism which is used to extend the operational capacities of the classification especially with respect to the accuracy and precision ratio. Moreover, systems designed and developed based on these techniques have relatively accurate decisions, which are basically informed, and then traditional models of classifications.

### 3.1. Artificial Neural Network

Artificial neural network (ANN) is an abstract expression of human brain neurons, which connect multiple neurons to form a variety of neural network models. Artificial neural network models consist of hidden layers, input layers, and output layers, each with a large number of neurons. Neurons are used in the hidden layer to simulate some complex linear functions for nonlinear classification. By increasing the number of hidden layers, the ability of nonlinear mapping can be enhanced.  Figure 1 illustrates the classical structure of an artificial neural network:

The input layer of the neural network uses the input layer to input the vector. Each component of the input vector is multiplied by the corresponding weight, and then the values are input to the hidden layer by linear overlay. In the hidden layer, the activation functions, such as hyperbolic tangent function and S-type function, are used to keep the nonlinear relationship between the input value and the output value, which enhances the expressive power of the model itself. The following is this mathematical expression:

(1) $$\begin{array}{c} \hat{y}=f\left(W•X+b\right). \end{array}$$

The upper form *W* represents the weight group, and the activation function and the input vector are represented by *F* and *X*, respectively. The artificial neural network algorithm loss function is defined by the following formula:

(2) $$\begin{array}{c} E\left(W\right)=\frac{1}{n}\sum_{i=1}^{n}{\left(y_{i},{\hat{y}}_{i}\right)}^{2}. \end{array}$$

The above formula ${\hat{y}}_{i}$ represents the estimated value of the parameter and *y_i_* represents the real value of the parameter. The loss function is used to obtain a set of *W* weights and reduce the loss function to the lowest value. The value of the loss function is inversely proportional to the accuracy of the model. The higher its value, the lower the accuracy.

RETRACTED

In the process of reverse propagation, neural network training employs the gradient descent approach to change weight W. It compares the real and predicted values of the neural network's output. There is a discrepancy between them. The loss function or other parameters can be utilized to compute gradient derivation in the direction of hidden layers, and mistakes are averaged allotted to each layer. This inaccuracy may be used by each layer of neurons to modify weight. In the mathematical terminology, this is the chain derivation rule. Iterate until the fault is identified, or halt the network model training if the number and duration of iterations fulfill the criteria.

### 3.2. Image Classification

Image classification uses the technology of applying classification technology to extract and classify target features. Pattern recognition uses computer technology to simulate human identification ability, that is, to describe, analyze, distinguish, and distinguish various things or objects by computer. Therefore, image classification is a recognition mode, and the process of classification is similar to that of pattern recognition.  Figure 2 shows the image recognition process, which preprocesses the input data on the image to improve the image quality, then extracts the key target areas after image segmentation, and finally extracts the target number features to classify using the corresponding best way.

#### 3.2.1. Image Preprocessing

In general, there are various kinds of interferences or worthless data in the original image. To filter the data by preprocessing, the valuable information in the data can be preserved and strengthened, the data redundancy can be reduced, and the convenience and reliability can be provided for further feature extraction. The operation modes are enhanced contrast, noise reduction, and sharpening.

RETRACTED

#### 3.2.2. Feature Extraction

There is a large amount of redundant image information in the image classification process. If this information is input directly into the image matrix, it will take a lot of memory space and reduce the computational efficiency. By extracting the image features with high recognition in the image, the data dimension can be reduced, the computational complexity of resources can be reduced, and the image feature vector classification effect in the classifier can be guaranteed.

#### 3.2.3. Classifier

In these models, classifier is the most basic but important and crucial task as if classification of the data values or object is carried out non seriously; then, it may cause certain problems like group may be compromised. Therefore, classifiers must be choosen intelligently keeping in view the requirement of issue under consideration. The classifier judges the sample type according to the feature vectors obtained during the input feature extraction stage in the image classification process. The classifier can be divided into supervised learning and unsupervised learning according to different learning methods. Unsupervised learning only enters sample characteristics into the classifier and does not make class labels for each sample, in order to find hidden structures in the label data. Supervised learning maps each training sample to its corresponding label, and the classifier adjusts parameters by comparing the real labels and classification labels on the features of the samples to judge the classification effect, and then feedback the final results.

### 3.3. Convolutional Neural Network

In-depth learning, in which the local and convolution kernels of the feature map are coupled, is a popular study topic in the field of machine learning. The convolution kernel weight parameters can be shared while generating each feature map, lowering the cost of constructing the convolution neural network. To perform the picture classification objective, the convolution neural network requires two procedures, as shown in Figure 3. First, the training pictures are used to create a convolution neural network classification model, which is then evaluated using the test image to determine the classification accuracy of the test set [18].

Forward propagation is used to extract image features. The steps required are sampling and convolution, and each image can only go from the input layer to the convolution layer, and the output is obtained using the activation function.

(3) $$\begin{array}{c} x^{l}=f\left(W^{l}x^{l}+b^{l}\right). \end{array}$$

The above formula *w* represents the weight, *l* represents the number of layers, *f* represents the activation function, and *b* represents the offset. During the forward propagation, a learnable convolution kernel convolutes multiple characteristic graphs in the upper layer and then uses the activation function to obtain a new characteristic graph.

(4) $$\begin{array}{c} x_{j}^{l}=f\left(\sum_{i\in M_{j}}X_{i}^{l-1}*k_{ij}^{l}+b_{j}^{l}\right). \end{array}$$

The upper *l* represents the current formation, the previous layer is represented by l−1, *X*_*j*_^1^ is the *j* feature map on the current layer, *k*_*ij*_^1^ is the convolution kernel between the *i* feature map on the current layer and the *j* feature map on the previous layer, and b*^l^_j_* is the offset value.

RETRACTED

After the convolution layer, the lower sampling layer can ignore the position changes such as rotation and tilt of the target, which can improve the robustness and performance of the algorithm, reduce the dimension of the feature graph, and reduce the problem of overfitting. The sampling layer is calculated by the following formula:

(5) $$\begin{array}{c} x_{j}^{l}=f\left(\beta_{j}^{l}\text{down}\left(x_{j}^{l-1}\right)+b_{j}^{l}\right). \end{array}$$

The downsampling function is represented by top down(). The weight of the convolution nucleus is updated via reverse propagation. Its essence is to compute the set sample label and forward propagation output value by error, and then utilise a range of techniques to acquire gradient values to update the convolution nucleus, such as pooling and convolution catheters. A loss function of local error operation is generally a square error loss function. The loss function of square difference may be stated as follows for solving multiple classification problems with *N* samples and *C* categories.

(6) $$\begin{array}{c} E^{N}=\frac{1}{2}\sum_{n=1}^{N}\sum_{k=1}^{C}{\left(t_{k}^{n}-y_{k}^{n}\right)}^{2}. \end{array}$$

The upper EN is the overall error of N samples, *t*_*k*_^*n*^ is the k-dimensional label corresponding to the *n* sample, and *y*_*k*_^*n*^ is the k-dimensional output corresponding to the *n* sample.

## 4. Artistic Painting Image Classification Based on Neural Network

Traditional image classification methods do not take the subjective characteristics of the paintings into account, but also extract the features manually. In the process of extracting the features, the generalization ability of the original heart model will be reduced and the features will be lost. Therefore, this paper puts forward a classification of art drawing images based on neural network, focusing on the optimization of network parameters and network structure design in the classification of art drawing images. By analyzing the problem that network structure depth affects classification performance, traditional series network structure can be obtained. Based on this, the convolution core size of each convolution layer can be set, and the convolution core size can affect the classification result, so as to optimize the network parameters. Then, a new convolution layer is paralleled between the two convolution layers to increase the network structure width, to achieve the purpose of combining multiple features, and to further optimize the network structure. By selecting a large number of different training samples, choosing Western and Eastern Painting image data collections to conduct experiments, the number of different training samples affects the classification results.

RETRACTED

### 4.1. Painting Image Classification Based on Artistic Style

It is vital to examine the age of the paintings, the style of the paintings, and the works of a particular artist when classifying the artistic styles of paintings. Image painting is a type of artificial work. Its key qualities include the artist's subjective sentiments, creative genre, and painting technique. As a result, classifying the creative styles of paintings is extremely challenging due to the requirement to communicate the artistic style features in a more comprehensive manner. The subjective sentiments of each artist are represented in the artistic style of painting, and some experts use the subjective object method to classify artistic styles of painting.

To solve this problem, a drawing image classification algorithm based on the rules of artistic style similarity is proposed. By analyzing western paintings and Dunhuang strokes, this algorithm analyzes the subjective characteristics of paintings. Image characteristics are difficult to describe a complete picture style, and there are great differences between local patch art styles. Therefore, it is proposed to divide a complete image into *M* × *N* local patches. Similarity between patches is calculated by the following formula:

(7) $$\begin{array}{c} G_{ij}=\frac{{\left|L_{i}-L_{j}\right|}^{2}}{\left(w_{i}\cdot h_{i}-1\right)}. \end{array}$$

*L_i_* represents the patch feature matrix on the first image. The height and width of the image patch are represented by *_i_* and *w*_*i*_, respectively. The formula is used to find the style similarity of this painting. Based on this, the Euclidean distance between similarity descriptors among images can be calculated, and then the similarity coefficients between images can be combined to form a similarity matrix, and AdaBoost is used as a classifier to classify the style of artistic works.

RETRACTED

### 4.2. Drawing Image Classification Based on Significance

Human beings have the ability to selectively or actively process visual information, the basic characteristics of human data. Bright colors on an image attract attention and are therefore called prominent colors, whereas areas of interest are prominent. Painting works are all formed by hand-drawn methods, so the artist's personal emotion will have a direct impact on the style of the work. Visual characteristics of human beings are obvious, and they will actively focus on the very obvious information in their paintings. This kind of image enhances people's attention, which is characterized by image prominence. Some experts have proposed using the matrix low rank decomposition method to extract the saliency features of paintings. The innovations of this method are that the saliency of transformable targets is an optimization problem, and the X-image matrix is decomposed into two parts: the saliency area and the nonsaliency area. The following is the calculation formula:

(8) $$\begin{array}{c} X={\text{XZ}}_{0}+E_{0}. \end{array}$$

*E *_0_ is the significant area in the formula and XZ_0_ is the nonsignificant area. The optimal solution of *E*_0_ and *Z*_0_ can be obtained by using Lagrange multiplier method after introducing some restrictions. Select multiple datasets here to verify the validity of the algorithm. The results show that there is ideal significance and image semantic classification is better.

## 5. Analysis of Fine Art Painting Image Classification Results

This section is dedicated to the extensive description and thorough analysis of the various results which are observed during the experimental setup. It is important to note that these results are based on actual values of the extensive analysis of dataset which are basically benchmark databases available online for extensive analysis and verification of the newly developed models.

### 5.1. Analysis of Comparing Result of Chinese Painting Dataset

This paper studies the classification of fine art drawing images based on neural network and puts forward a variety of above neural network-based algorithms to extract fine art drawing images. An ArtDimage is created here to test the classification effect of fine art drawing images. The total number of images stored in this dataset is 60,000, which is divided into 100 categories. The number of images in each class is 600. This dataset is a Chinese Art Painting dataset and trains the relational network model to complete data classification tasks.

RETRACTED

The main types of Chinese Art Painting image data collection are flowers and birds, mountains and rivers, and people. When the task on the ArtDimage training set is 3-way, 5-shot, that is, which of the three types is randomly selected each time in the ArtDimage training set. There are 5 training graphics in each type and 15 test images in total. When classifying the image data collection of Chinese fine art drawing, five training images from three different types of flower, bird, landscape, and person are extracted, and 15 total training images are obtained. After calculation, the classification accuracy can be obtained. In this way, the image classification results under 3-way, 20-shot, 3-way, 50-shot tasks will be affected by the addition of training datasets to the model classification accuracy test. The training iterations for each task on the ArtDimage dataset are as many as 80,000. The pretraining model for each task is used to test drawing data. To test 600 times for each task, select a confidence interval with an accuracy of up to 95% and set the learning rate to 0.001. The experimental results are listed in Table 1.

The data in Table 1 shows that the accuracy rate of training 3-way and 50 shot tasks is 66.7%, that of training 30-way and 20 shot tasks is 72.4%, and that of training 0-way and 50 shot tasks is 78%. Therefore, when there is a large dataset in the training task, the corresponding test accuracy is high. Therefore, training a large number of labeled Chinese art painting datasets through neural network can obtain an accuracy of 95.68%.

The experimental configuration and task on the Chinese art painting dataset are exactly the same. The 3-way and 5-shot tasks are trained again on the pretraining Dunhuang mural dataset, with up to 600 iterations and 60 iterations at a time. The accuracy results of this experiment are saved. The final results are shown in Figure 4 [19].

Analyze the data in Figure 4, in which the abscissa is the number of iterations and the ordinate is the accuracy of this test. In the Dunhuang mural dataset, the average accuracy of 3-way and 5-shot tasks fluctuates around 65%. This paper tests 300 Dunhuang mural datasets based on the neural network model, and the accuracy is 70%, which shows that the accuracy of this model is high.

### 5.2. The Influence of the Number of Training Samples on the Classification Results

The amount of training samples has a direct impact on the convolutional neural network's classification performance. There will be an overfitting problem if there are few training samples. Using two datasets, the Oriental painting image and the western painting image, this research investigates how the amount of training samples influences classification outcomes. Select 100, 200, 300, 400, 500, and 600 photos at random as training samples from the three types of figures, flowers and birds, and landscape in Oriental art images, and then 200 images at random as test samples from the remaining samples. Images in western paintings are classified into two categories: landscape and character. Similarly, 50, 100, 150, 200, 250, 300, and 350 images are selected as training samples, and then 150 images in the remaining samples are randomly selected as test samples. In this paper, the convolution neural network structure of the optimized Oriental painting image dataset and the western painting image dataset is used, and the accuracy results of Oriental painting image training classification are shown in Figure 5, and the accuracy of Western painting image classification is shown in Figure 6 [20, 21].

RETRACTED

According to the data in Figure 5, when the number of Oriental painting image training samples is 100, 200, 300, 400, 500, and 600 images, respectively, the corresponding classification accuracy is 67.6%, 74%, 88.9%, 92.6%, 93.5%, and 94.6%. After increasing the number of training samples, the classification accuracy of convolutional neural network model is also gradually improved.

By analyzing the data in Figure 6, when the number of Western painting image training samples is 50, 100, 150, 200, 250, 300, and 350 images, the corresponding classification accuracy is 88.9%, 93.2%, 94.6%, 95.7%, 97%, 96.5%, and 98%. With the continuous increase of the number of training samples, the image accuracy of the optimized neural network model is also increasing. The above results are due to the fact that the neural network belongs to the deep network structure, which contains multiple hidden layers, which can strengthen the feature learning ability of the convolutional neural network. Therefore, continuously increasing the number of training samples can fully reflect the feature learning ability of neural network, and the learning features can better express the data and improve the classification accuracy.

### 5.3. The Results of This Method Compared with Those of CNN, NN, and DBN

In this paper, the same dataset is selected to test the performance of the proposed algorithm, DBN, NN, and CNN algorithms. 780 images are randomly selected from the sample set of characters, landscapes, flowers and birds, and the remaining 20 images are used as the test set. The classification results obtained by different depth algorithms are listed in Table 2.

By analyzing the data in Table 2, it can be seen that the algorithm in this paper and NN, CNN, and DBN can greatly improve the recognition rate of learning algorithm. Compared with the other three methods, the algorithm in this paper has strong classification performance. The convergence steps of the comparison algorithm, NN, CNN, and DBN algorithm are 171, 221, 200, and 200, respectively. The algorithm with the smallest convergence steps is the algorithm in this paper, so the classification performance is stronger.

RETRACTED

## 6. Conclusion

Classification is defined as the process of separating various objects in to the classes or groups where probability of similarity indexes between elements of a particular group is very high, i.e., it is high likely that elements or objects or data belong to a group which will be similar than other data values belonging to other groups or classes. Art painting image classification is the most difficult part of image classification. Because there are many types of painting images and there are great differences between Oriental painting and Western painting, it needs a lot of data calculation. However, the traditional feature extraction methods cannot extract more information, and the speed is slow and the accuracy is low. Therefore, this paper uses neural network algorithm in the study of art painting image classification. Firstly, the painting image classification algorithm based on art style is used to analyze and process the painting image art style, and calculate the similarity of each art painting image. Then, the image semantics is classified by the painting image classification algorithm based on significance. According to the above two algorithms, the art painting images are classified, and the classification effect is ideal and the accuracy is high. At the same time, the dataset verification method is used to test the effect of this method on the classification of art painting images. The results show that this algorithm is feasible.

## Figures and Tables

**Figure 1:** Structure diagram of artificial neural network.

**Figure 2:** Image recognition process.

**Figure 3:** Image classification algorithm flow based on convolution neural network.

**Figure 4:** Accuracy analysis of Dunhuang mural dataset.

**Figure 5:** Oriental painting image training classification accuracy.

**Figure 6:** Accuracy of Western painting image classification.

**Table 1:** Comparison of the classification accuracy of different training datasets.

Training dataset	3-way, 50-shot (%)	30-way, 20-shot (%)	30-way, 50-shot (%)
Accuracy rate (%)	66.7	72.4	78

**Table 2:** Comparison of the classification results of different depth learning algorithms.

Algorithm type	Training data set	Average accuracy (%)	Convergence steps	Training time (s)
Neural network	2340	67.4	171	944.5
CNN	2340	66	200	897.2
NN	2340	79	221	30.5
DBN	2340	61.5	200	30.2

RETRACTED

## Data Availability

The datasets used and/or analyzed during the current study are available from the corresponding author on reasonable request.
